This article has been retracted.

# Numb inhibits epithelial-mesenchymal transition via RBP-Jκ-dependent Notch1/PTEN/FAK signaling pathway in tongue cancer

**DOI:** 10.1186/s12885-019-5605-5

**Published:** 2019-04-25

**Authors:** Jin-Yun Li, Wen-Xiao Huang, Xiao Zhou, Jie Chen, Zan Li

**Affiliations:** Department of Head and Neck Surgery, Hunan Cancer Hospital and Affiliated Cancer Hospital of Xiangya School of Medicine, Central South University, No.283, Tongzipo Road, Yuelu District, Changsha, 410013 Hunan Province People’s Republic of China

**Keywords:** Tongue squamous cell carcinoma (TSCC), Numb, Notch1 signaling, PTEN, Epithelial-mesenchymal transition (EMT)

## Abstract

**Background:**

Oral cancer has been estimated as the sixth most frequent solid cancer all over the world, in which tongue squamous cell carcinoma (TSCC) is the most common type of oral cancers. However, the mechanism of TSCC metastasizing to lymph node and distant sites has not been completely understood.

**Methods:**

In this study, RT-qPCR method was used to detect the mRNA level of Numb, PTEN and Notch1 genes, as well as EMT-associated genes. Western blot assay was utilized to detect protein level of these genes. In addition, we determined cell proliferation by MTT assay and employed transwell invasion assay and wound healing assay to probe the abilities of invasion and migration, respectively. To investigate the role of PTEN, its inhibitor VO-Ohpic trihydrate was used to treat SCC-4 and CAL27 cells.

**Results:**

We found that Numb expression was downregulated in SCC-9 and CAL-27 cells compared to NHOK cells. Instead, Notch1 level in SCC-9 and CAL-27 cells were higher than that in NHOK cells. Furthermore, the results showed that Numb overexpression significantly suppressed proliferation, migration and invasion of SCC-9 and CAL-27 cells via regulating Notch1 signaling and EMT-related genes expression. By contrast, we observed that RBP-Jκ knockdown had an inhibitory role in proliferation, migration and invasion of SCC-9 and CAL-27 cells. In cells with Numb overexpression or RBP-Jκ knockdown, p-FAK and EMT-related genes were remarkably regulated.

**Conclusions:**

Our findings provide new mechanism of understanding the metastasis of TSCC and help develop therapeutic strategies for treating tongue cancer.

## Background

Oral cancer accounts for about 1–3% of all human cancer cases, which is the 6th most occurred cancer in the world. Tongue squamous cell carcinoma (TSCC) is the most common type of oral cancer [1–3]. Most importantly, lymph node and distant metastasis are the most adverse prognostic factors and will cause the death of TSCC patients [4, 5]. In spite of large advances in understanding how tongue cancer initiates and progresses, the number of deaths of TSCC patients increased by approximately 10% over the past 5 years [6, 7]. Thus, it remains urgent to further clarify the molecular mechanism of carcinogenesis and metastasis of tongue cancer.

The Notch1 signaling pathway is an evolutionarily conserved pathway, which has been involved in a wide variety of physiological and pathological processes, including cell fate determination, cell differentiation, tissue patterning and morphogenesis, and various types of cancer [8–10]. It has been studied that Notch1 signaling pathway participates in invasion of TSCC via regulating matrix metalloproteinases (MMPs) [11]. Therefore, we attempted to figure out the detailed mechanism of how Notch1 signaling and its regulators (like Numb) contributes to progression and metastasis of tongue cancer.

Phosphatase and tensin homolog (PTEN), commonly regarded as the tumor suppressor, is reported to regulate cancer cell invasion through blocking a variety of signaling pathways [12, 13]. In TSCC tissue, PTEN expression was lower than that in noncancerous counterparts, which suggested PTEN might act as tumor suppressor of TSCC [14, 15]. More intriguingly, Siming Xie et al. reported that PTEN upregulation suppresses invasion of tongue cancer cells through repression of EMT, which provided direct evidence that PTEN played tumor inhibitory role in progression and metastasis of tongue cancer [16].

Here, we reveal Numb, negative regulator of Notch1 signaling pathway, plays an inhibitory role in EMT of tongue cancer cells via regulating Notch1/RBP-Jκ/PTEN/p-FAK axis. In this study, we confirmed the crucial role of RBP-Jκ in EMT of tongue cancer cells. We believed that these findings will facilitate the development of targeted drugs used for treating tongue cancer.

## Methods

### Cell lines and reagents

Tongue squamous cancer cell lines (SCC-9 and CAL-27) and 293 T cell were from American Tissue Culture Collection (ATCC, USA) and cultured in Dulbecco’s Modified Eagle’s Medium (DMEM, Hyclone) with 10% fetal bovine serum (FBS) and 100 U/mL penicillin/streptomycin at 37 °C, 5% CO_2_. Of which, SCC-9 cells were grown in 1:1 Hams F-12, DMEM (modified). Primary normal human oral keratinocytes (NHOK), purchased from PriCells, were isolated from human gingival tissues and cultured as described previously [17]. PTEN inhibitor VO-Ohpic trihydrate was purchased from MedChemExpress (USA) and worked at the concentration of 35 nM.

### Plasmid and lentivirus packaging

Numb cDNA sequence was cloned and ligated into pCDH-MCS-EF1-puro vector. RBP-Jκ short hairpin RNA (shRNA-RBP-Jκ) or negative control shRNA (shRNA-NC) were inserted into PLKO.1 vector. In order to make lentiviruses, pPAX2 and pVSVG vectors plus transfer vector were introduced into 293 T cells. Then, we harvested the supernatant at 48 h post transfection, which was filtered with 0.45 μm membrane and concentrated by a centrifugal filter (EMD Millipore, Amicon Ultra 100 k). When subject to virus infection, the cells medium was treated with virus supernatant at 1:5 ratios, post 24 h, we used ~ 2 μg/mL puromycin to select the Numb-overexpressed stable cell lines. The shRNA sequences are synthesized as previously described [18].

### Western blot

We performed this experiment as standard procedure in accordance with previous descriptions [8]. The following antibodies were used: anti-E-cadherin (cell signaling technology, USA), anti-N-cadherin (cell signaling technology, USA), anti-Snail (cell signaling technology, USA), anti-MMP-9 (cell signaling technology, USA), anti-Numb (cell signaling technology, USA), anti-Notch1 (cell signaling technology, USA), anti-FAK (cell signaling technology, USA), anti-p-FAK (cell signaling technology, USA), anti-PTEN (cell signaling technology, USA), anti-RBP-Jκ (millipore, USA), anti-GAPDH (Proteintech, USA).

### Invasion assay

To perform this assay, TSCC (1 × 10^5^cells) were mixed with about 200 μL of FBS-free medium. Chambers containing 8.0 μm pore membranes (Millipore) with matrix was used in this assay. The TSCC cells were seeded into the top chamber. Afterwards, about 500 μL complete medium was added to bottom chamber. Roughly 48 h post incubation, the invaded cells were fixed and stained with crystal violet, and finally were counted using the inverted microscope.

### Wound healing assay

We measured migration of cells in vitro through wound healing assay. In brief, 2 × 10^5^ SCC-9 and CAL-27 cells were passaged to 6-well plates. The cells were incubated in the complete culture medium under normal conditions for 16 h. then, we scratched the monolayer and incubated cells in fresh medium without FBS for 24 h. Eventually, we measured the wound width. we visualized and photographed 3 different locations under the inverted microscope.

### RT-qPCR

We harvested cells and extracted total RNAs by Trizol method. Then, chloroform was added to the solution. The sample was subject to centrifuge at 12,000 rpm for 10 min, and was transferred to new RNase-free EP tube. Resulting solution was mixed with equal volume of isopropanol and subject to centrifuge at 12,000 rpm for 10 min. After that, removing the supernatant and adding 70% ethanol to wash pellet. Eventually, discarding the ethanol and drying the RNA pellet. And, we used 35 μL Rnase-free H_2_O to dissolve RNA.

We employed ~ 1 μg of RNA for reverse transcription. SYBR dye was used to detect signaling, the GAPDH serves as internal control. The primers used in this study as follows:

- Numb-F: TCTGCTCCGATGACCAAACC
- Numb-R: GCACCAGAAGATTGACCCCA
- Notch1-F: CAACTGCCAGAACCTTGTGC
- Notch1-R: GGCAACGTCAACACCTTGTC
- GAPDH-F: GAGTCAACGGATTTGGTCGT
- GAPDH-R: TTGATTTTGGAGGGATCTCG

### Statistical analysis

All experiments were conducted for three replicates, all values were represented as mean ± SD, comparisons of two groups were done using two-tailed unpaired student’s *t*-test. *P < 0.05 was considered statistically significant.

## Results

### Numb and Notch1 expressions were altered in tongue squamous cancer cell lines

Recently, it has been studied that Notch1 signaling is implicated in progression of tongue cancer [8]. To validate, we examined the expression of Numb (Notch1 regulator) and Notch1 in tongue squamous cancer cell lines (SCC-9 and CAL-27) and normal human oral keratinocytes (NHOK) by RT-qPCR method. We found that Numb expression level was significantly decreased in SCC-9 and CAL-27 cells compared with that in NHOK cells (Fig. 1a). By contrast, the level of Notch1 was increased by about 2 folds in SCC-9 and CAL-27 cells (Fig. 1b). These data suggested that, indeed, Numb and Notch1 signaling were implicated into tongue cancer progression.

**Fig. 1:** Expression of Numb and Notch1 in tongue cancer cell lines (CAL-27 and SCC-9) and normal human oral keratinocytes (NHOK). **a** RT-qPCR analysis shows the level of Numb in SCC-9, CAL-27 and NHOK cells. **b** RT-qPCR analysis shows mRNA level of Notch1 in SCC-9, CAL-27 and NHOK cells. The data were represented as mean ± SD from 3 biological replicates (*p < 0.05; **p < 0.01)

### Numb overexpression inhibits proliferation, invasion and migration of SCC-9 and CAL-27

To further confirm the anti-tumor role of Numb in tongue cancer, we constructed Numb-overexpressed SCC-9 and CAL-27 cell lines. First, we used MTT assay to evaluate SCC-9 and CAL-27 cells growth and found that cell proliferation ability of cells were markedly suppressed upon Numb overexpression compared to negative control (NC) (Fig. 2a).

**Fig. 2:** Numb overexpression inhibits proliferation, invasion and migration of SCC-9 and CAL-27 cells. **a** Cell proliferation assay and quantification of NC (mock) or Numb-overexpressed SCC-9 and CAL-27 cells by MTT assay at 48 h after transfection. NC denotes cells transfected with empty vector, Numb denotes cells transfected with pCDH-Numb. **b** and **c** Wound healing assay and quantification shows the migration ability of NC (mock) or Numb-overexpressed SCC-9 and CAL-27 cells. The photographies were taken at the time points of 0, 24, 48 h. Magnification × 10(5000 μm) in wound healing assay. **d** and **e** Transwell assay and quantification shows the invasion ability of NC (mock) or Numb-overexpressed SCC-9 and CAL-27 cells. The photographies were taken at 24 h. Magnification× 50(2000 μm) in transwell assay. The data were represented as mean ± SD from 3 biological replicates (*p < 0.05; **p < 0.01; ***p < 0.001)

Next, we assessed cell migration by wound healing assay when the cells transfected with empty vector or Numb at the time points of 0, 24, 48 h. The results demonstrated that Numb-overexpressed SCC-9 and CAL-27 cells displayed impaired migration ability relative to NC group cells (Fig. 2b and c). In addition, we also investigated the role of Numb in invasion of tongue cancer cells (SCC-9 and CAL-27) using transwell invasion experiment at 24 h. Our data revealed that the number of invaded tongue cancer cells expressing Numb was remarkably lower than NC group cells (Fig. 2d and e). Collectively, these results indicated that Numb had an inhibitory role in tongue cancer proliferation and metastasis.

### Numb regulates Notch1 signaling and EMT-associated genes expression

In order to dissect the molecular mechanism Numb-suppressed proliferation and tongue cancer cells EMT, we probed expression of Notch1 and EMT-associated genes (Fig. 3a and b). Western blot analyses demonstrated that Notch1 expression level was decreased in Numb-overexpressed SCC-9 and CAL-27 cells. More importantly, we observed that EMT-inhibited genes (E-cadherin) expression level was upregulated, whereas RBP-Jκ and EMT-promoted genes (N-cadherin, Snail, MMP-9) expression level was downregulated. These data showed Numb had a critical role in regulation of Notch1 signaling, RBP-Jκ and EMT-associated genes expression, which is more likely to mediate Numb-inhibited EMT of tongue cancer cells.

**Fig. 3:** Numb reduces Notch signaling- and EMT-associated genes expression. **a** Western blot analyses shows protein levels of Numb, Notch1, RBP-Jκ and EMT-related genes (E-cadherin, N-cadherin, Snail-1, MMP-9) in mock or Numb-overexpressed SCC-9 and CAL-27 cells. GAPDH acts as internal control. **b** Gray level analysis of the protein levels of Numb, Notch1, RBP-Jκ and EMT-related genes (E-cadherin, N-cadherin, Snail-1, MMP-9) in mock or Numb-overexpressed SCC-9 and CAL-27 cells after western blot. The mean ± SD in the graph represents the average levels from three replicates. *p < 0.05, **p < 0.01, ***p < 0.001

### PTEN inhibition leads to increased expression of EMT-associated genes expression

To explore the role of PTEN in regulation of EMT-associated genes expression in tongue cancer cell lines (SCC-9 and CAL-27), we utilized PTEN inhibitor VO-Ohpic trihydrate to abolish the function of PTEN and then detected expression level of EMT-associated genes (Fig. 4a and b). As shown in the western blot, PTEN expression was suppressed by VO-Ohpic trihydrate in Numb-overexpressed SCC-9 and CAL-27 cells. However, phosphorylated form of FAK was elevated in the presence of VO-Ohpic trihydrate. In addition, the result showed VO-Ohpic trihydrate treatment disrupted EMT-related genes expression level modulated by Numb. Together, our data suggested that PTEN inhibitor VO-Ohpic trihydrate could effectively block Numb-inhibited EMT genes expression in SCC-9 and CAL-27 cells.

**Fig. 4:** PTEN inhibition results in increased expression of EMT-associated genes expression. **a** Western blot analyses showing the protein level of PTEN, FAK, p-FAK and EMT-related genes (N-cadherin, E-cadherin, Snail-1, MMP-9) in mock, Numb-overexpressed, Numb-overexpressed plus VO-Ohpic trihydrat-treated SCC-9 and CAL-27 cells. GAPDH serves as internal control. **b** Gray level analysis of the protein level of PTEN, FAK, p-FAK and EMT-related genes (N-cadherin, E-cadherin, Snail-1, MMP-9) in mock, Numb-overexpressed, Numb-overexpressed plus VO-Ohpic trihydrat-treated SCC-9 and Cal-27 cells after western blot. The mean ± SD represents the average levels from 3 replicates. *p < 0.05, **p < 0.01, ***p < 0.001

### RBP-Jκ-depleted tongue cancer cells exhibits attenuated proliferation, invasion and migration

Next, we attempted to assess whether RBP-Jκ was key for proliferation and metastasis of tongue cancer cells. We generated RBP-Jκ-depleted tongue cancer cell lines (SCC-9 and CAL-27) using short hairpin RNA approach. Then, MTT experiment was carried out to detect cell proliferation of SCC-9 and CAL-27 cells. We found that RBP-Jκ knockdown SCC-9 and CAL-27 cells grew more slowly than NC cells (Fig. 5a).

**Fig. 5:** RBP-Jκ-depleted tongue cancer cells exhibits attenuated proliferation, invasion and migration. **a** Cell proliferation assay and quantification of NC (sh-NC) or RBP-Jκ-knockdown (RBP-Jκ shRNA) SCC-9 and CAL-27 cells by MTT assay at 48 h after transfection. **b** and **c** Wound healing assay and quantification shows the migration ability of NC (sh-NC) or RBP-Jκ-knockdown (RBP-Jκ shRNA) SCC-9 and CAL-27 cells. The photographies were taken at different time points of 0, 24, 48 h. Magnification × 10(5000 μm) in wound healing assay. **d** and **e** Transwell invasion assay and quantification shows the invasion ability of NC (sh-NC) or RBP-Jκ-knockdown (RBP-Jκ shRNA) SCC-9 and CAL-27 cells. The photographies were taken at 24 h. The photographies were taken at 24 h. Magnification× 50(2000 μm) in transwell assay. The data were represented as mean ± SD from 3 biological replicates (*p < 0.05; **p < 0.01)

To test whether RBP-Jκ had a role in invasion and migration of tongue cancer cells, we carried out transwell invasion assay and wound healing assay to evaluate the invasion and migration ability of the cells, respectively. We observed that RBP-Jκ knockdown resulted in impaired migration capability of SCC-9 and CAL-27 cells (Fig. 5b and c). In parallel, fewer numbers of invaded cells (decreased by 30–40%) were stained by crystal violet when the cells were transfected with RBP-Jκ shRNA compared to NC cells at 24 h (Fig. 5d and e). In summary, all these results revealed that RBP-Jκ was important for proliferation, migration and invasion of tongue cancer cells (SCC-9 and CAL-27).

### RBP-Jκ knockdown regulates PTEN and EMT-associated genes expression

To clarify the underlying molecular mechanism of RBP-Jκ knockdown-caused proliferation and metastasis change of tongue cancer cells, we attempted to probe PTEN, FAK and EMT-related genes expression after RBP-Jκ knockdown in SCC-9 and CAL-27 cells (Fig. 6a and b). Western blot analyses demonstrated that PTEN and EMT-inhibited gene (E-cadherin) expression level were upregulated in RBP-Jκ knockdown cells, on the other hand, p-FAK and EMT-promoted genes (N-cadherin, Snail, MMP-9) expression level was downregulated upon RBP-Jκ depletion. Therefore, we concluded that RBP-Jκ was a key regulator of PTEN/FAK/EMT-related genes pathway.

**Fig. 6:** RBP-Jκ knockdown regulates PTEN and EMT-associated genes expression. **a** Western blot analyses showing the protein level of PTEN, FAK, p-FAK, RBP-Jκ and EMT-related genes (N-cadherin, E-cadherin, Snail-1, MMP-9) in NC (sh-NC) or RBP-Jκ-knockdown (RBP-Jκ shRNA) SCC-9 and CAL-27 cells. GAPDH serves as internal control. **b** Gray level analysis of the protein level of Numb, Notch1, RBP and EMT-related genes (E-cadherin, N-cadherin, Snail-1, MMP-9) in mock or Numb-overexpressed SCC-9 and CAL-27 cells after western blot. The mean ± SD represents the average levels from 3 replicates. *p < 0.05, **p < 0.01

### PTEN inhibition leads to increased expression of EMT-associated genes expression with abatement of RBP-Jκ

We next attempted to figure out whether PTEN inhibitor also influenced expression of p-FAK and EMT-related genes in the tongue cancer cells with RBP-Jκ knockdown (Fig. 7a and b). Western blot analyses showed PTEN and E-cadherin was modestly downregulated in RBP-Jκ-knockdown cells treated with VO-Ohpic trihydrate. Nonetheless, p-FAK and EMT-promoted genes (N-cadherin, Snail, MMP-9) expression level were modestly upregulated in response to VO-Ohpic trihydrate treatment. Our data indicated that PTEN inhibition had the ability to partially rescue RBP-Jκ knockdown-induced changes in expression of p-FAK and EMT-regulated genes.

**Fig. 7:** PTEN inhibition leads to increased expression of EMT-associated genes expression in the absence of RBP-Jk. **a** Western blot analyses showing the protein level of PTEN, FAK, p-FAK and EMT-related genes (N-cadherin, E-cadherin, Snail-1, MMP-9) in NC (sh-NC), RBP-Jκ-knockdown (RBP-Jκ shRNA), RBP-Jκ-knockdown (RBP-Jκ shRNA) plus VO-Ohpic trihydrat-treated SCC-9 and CAL-27 cells. GAPDH acts as internal control. **b** Gray level analysis of the protein level of PTEN, FAK, p-FAK and EMT-related genes (N-cadherin, E-cadherin, Snail-1, MMP-9) in NC (sh-NC), RBP-Jκ-knockdown (RBP-Jκ shRNA), RBP-Jκ-knockdown (RBP-Jκ shRNA) plus VO-Ohpic trihydrat-treated SCC-9 and CAL-27 cells. The mean ± SD represents the average levels from 3 replicates. *p < 0.05, **p < 0.01

## Discussion

Recently, Notch1 has been shown to exert its oncogenic role in various types of cancers, including lung, colorectal, T-cell acute lymphoblastic leukemia, breast and prostate carcinomas [19, 20]. However, the detailed mechnism by which Notch1 regulates progression and metastasis of tongue cancer remains unclear. Indeed, Notch1 signaling is activated in human tongue carcinoma [21]. In our study, we reveal the critical role of Numb and RBP-Jκ in regulating EMT of SCC-9 and CAL-27 cells, thereby highlighting the existence of Numb/Notch1/RBP-Jκ/PTEN/FAK/EMT axis in tongue cancer cells.

Epithelial-mesenchymal transition (EMT), a key prerequisite for individual development and cancer cells metastasis, can be initiated or controlled by developmental and various environmental cues [22]. In breast and other cancers, Notch1 signaling induced EMT phenotype by upregulating EMT-promoted genes (Slug and Snail) expression, then downregulated E-cadherin [23, 24]. Consistent with previous studies, we observed that Notch1 also had the ability to regulate EMT-related genes expression in tongue cancer cells. In addition, we found Notch1 influenced EMT of tongue cancer through its downstream effector PTEN and RBP-Jκ. These results provided more insight into the mechanism of Notch1-induced EMT.

Numb is the human homologue of the protein numb, initially discovered in *Drosophila melanogaster*, well-known for its multifaceted role in neurogenesis [25]. The antagonistic role of Numb in the Notch1 pathway led researchers to investigate the potential role of Numb in tumorigenesis in a number of tumors [26]. However, to date, little is known about whether Numb had an effect on EMT of tongue cancer cells. Our study, for the first time, investigate and clarify the inhibitory role of Numb in proliferation, invasion and migration of tongue cancer cells through negatively regulating Notch1 signaling and modulating EMT-related genes expression.

In order to elucidate the downstream mechanism of Notch1-induced EMT of tongue cancer, we focused on tumor suppressor PTEN, a reported target of Notch1 via CBP-1 binding to PTEN DNA promoter [27]. It is well established that PTEN loss is a prognostic marker and contributes to development of tongue cancer [28]. We also confirmed the critical role of *PTEN* in Numb overexpression- and RBP-Jκ knockdown-caused changes in proliferation and metastasis of tongue cancer cells by employing PTEN inhibitor VO-Ohpic trihydrate. Besides, we further explored and confirmed that PTEN exerted its role through regulating the activity of FAK (p-FAK level), thereby affecting expression of EMT-associated genes.

## Conclusions

In summary, we propose that Numb, negative regulator of Notch1 signaling, plays a suppressive role in proliferation and metastasis of tongue cancer cells. Mechanistically, Notch1 further regulates PTEN via in a RBP-Jκ-dependent manner to impact activity of FAK that is essential for EMT phenotype of tongue cancer cells. Nonetheless, the further investigation of FAK importance in EMT of tongue cancer cells requires to be undertaken by using FAK inhibitor or shRNA.

## Abbreviations

EMT: Epithelial-mesenchymal transition
FBS: Fetal bovine serum
MMPs: Matrix metalloproteinases
NC: Negative control
NHOK: Normal human oral keratinocytes
PTEN: Phosphatase and tensin homolog
TSCC: Tongue squamous cell carcinoma
